The article "Preparation of Iron Oxide and Titania-Based Composite, Core-Shell Populated, Nanoparticulates Material by Two-Step LASER Ablation in Aqueous Media as Antimicrobial and Anticancer Agents" was retracted in 2023. Reasons: signs of a paper mill; compromised peer review; unreliable results or conclusions.

# Preparation of Iron Oxide and Titania-Based Composite, Core-Shell Populated, Nanoparticulates Material by Two-Step LASER Ablation in Aqueous Media as Antimicrobial and Anticancer Agents

**DOI:** 10.1155/2022/1854473

**Published:** 2022-01-25

**Authors:** Hasan H. Bahjat, Raid A. Ismail, Ghassan M. Sulaiman, Hamdoon A. Mohammed, Mohsen Al-Omar, Salman A. A. Mohammed, Riaz A. Khan

**Affiliations:** ^1^Division of LASER Science and Technology, Department of Applied Sciences, University of Technology, Baghdad 10066, Iraq; ^2^Division of Biotechnology, Department of Applied Sciences, University of Technology, Baghdad 10066, Iraq; ^3^Department of Medicinal Chemistry and Pharmacognosy, College of Pharmacy, Qassim University, Qassim 51452, Saudi Arabia; ^4^Department of Pharmacognosy, Faculty of Pharmacy, Al-Azhar University, Cairo 11371, Egypt; ^5^Department of Pharmaceutical Chemistry and Pharmacognosy, College of Pharmacy, JUST, Irbid, Jordan; ^6^Department of Pharmacology and Toxicology, College of Pharmacy, Qassim University, Qassim 51452, Saudi Arabia

## Abstract

Iron oxide and titania-based composite nanoparticles (NPs) populated with core-shell structures, as part of the mixture of the monometallic NPs, were prepared in water medium by the two-fluence LASER ablation technique by applying 30 and 60 mJ/cm^2^ LASER energy irradiations. The prepared monometallics, composite, and core-shell NPs structures were confirmed from the XRD, TEM, and EDX analyses, followed by the FE-SEM and UV absorptions. Optically, the NPs exhibited an increase in the energy gap from 3.27 eV to 3.75 eV as LASER fluence increased from 30 mJ/cm^2^ to 60 mJ/cm^2^. The average NPs core size distributions for the core-shell material ranged at ∼70 nm with the shell thickness around 20 nm. The biggest NPs were of ∼170 nm size which were sparsely distributed. The magnetization behaviors of the NPs were also investigated using the vibrating sample magnetometer (VSM). The NPs showed antimicrobial activities against the pathogenic species: *Escherichia coli* and *Staphylococcus aureus*. The antimicrobial activities of the synthesized NPs, synthesized under the influence of magnetic fields, were found to be more potent than the NPs synthesized without the presence of any magnetic field. The NPs prepared under the influence of the magnetic fields also comparatively exhibited higher levels of cytotoxicity against lung cancer cell lines (A549) than the NPs prepared under no magnetic field's influence by the similar energy level effects of the LASER fluence. The flow cytometry analyses confirmed the NPs' cytotoxic impacts against the human lung cancer A549 cell lines through the initiation of apoptosis and promotion of the cell cycle arrest at the G1 phase of cell division. To further confirm the cytotoxic effects and the mechanism of the anticancer activity of the synthesized NPs against the A549 cell lines, several related parameters (cell viability, membrane permeability, nuclear intensity, and cytochrome-C release) were analyzed using the high-content screening (HCS) assay. The study suggested that the prepared NPs have potential as antimicrobial and also as anti-lung-cancer agents as tested *in vitro*. These NPs can also be part of combined chemotherapy in different oncological interventions, as well as a sonosensitizer in sonomagnetic heating-based therapy, especially for cancers.

## 1. Introduction

Nanotechnology deals with the process of synthesizing materials that are different in size, shape, chemical composition, characteristics, and reactivity. Their sizes range between 1 and 100 nm. The nanoparticles (NPs) are among the major nanomaterials produced from metallic and nonmetallic sources that are employed in diverse applications in different fields including medicine, optoelectronics, and catalysis [1, 2]. Due to size-dependent properties, the noble metal NPs, for example, gold and silver, exert important functions in biology, medicine, and electronics. Structurally, the NPs are characterized by a high surface-to-volume ratio, which confers them with higher catalytic and other responsive properties [3].

The metal oxide-based nanomaterials of nanocomposite nature have been produced by employing various methods of synthesis, the majority of which rely on hazardous chemical processing that renders the synthetic protocol environmentally challenging, costly, and harmful to living creatures' health [3]. For these reasons, the necessity to minimize the usage of toxic chemicals in preparation is imminent, and the development of effective, simpler, and safer methods are continuously sought. Based on these understandings and the context for a benign method of NPs preparations, the pulsed LASER ablation technique was developed as a preferred tool to synthesize nanocomposites, wherein the compression of the metallic targets is achieved under liquid media [4]. The approach is feasible owing to its feasibility to handle, its efficiency, and environmentally safe nature. The method has been extensively employed in the synthesis of colloidal solutions of extensive arrays of NPs in a number of liquid media, and as a result, the NPs with a variety of shapes have been produced and successfully utilized in numerous biomedical applications [5].

The current approach targets the preparation of antimicrobial agents with a particular focus on the high-infectious bacteria that pose a global threat to millions of the population annually [6, 7]. As part of the traditional practice for reducing and containing various infections, high doses of several classes of antibiotics are prescribed. Nonetheless, the bacteria and other pathogenic microorganisms have consistently responded with genetic mutations that have enhanced their resistance, and it has proved the futility of several antimicrobial agents [8, 9]. To combat the infections, there has been a continuous development of various compounds and materials that include quaternary ammonium compounds [10], carbon nanotubes [11], metal-ions formulations [12], metal-oxide molecules [13], and noble metal-based materials [14]. Such materials, notwithstanding, exert multiple downside effects as complex environmental pollutants that require high costs for their removal as part of the extraction of the toxic nanosubstrates to eliminate the polluting effects [8]. Therefore, the urge to develop novel agents with high antimicrobial properties have been continuously pursued. Furthermore, another serious and uninterrupted threat to human health is posed by the occurrences of various forms of cancers, and with over eleven million new cases being registered annually, and the situation is alarming [15]. Interestingly, the cancer cells also possess the potential to resist chemotherapy, and they also exhibit multidrug resistance (MDR) to treatments. To improve the efficacy of cancer therapy and bring the oncological chemotherapy-generated side effects to a minimum, different types of treatments modules have been reconnoitered. The advances in materials science and the emergence of nanotechnology have led to remarkable improvements in the synthesis of materials with unique properties that also exhibit feasible drug delivery preferences. These nanotechnology-based products as potent materials and compounds have improved the delivery and have propelled to achieve newer levels of antitumor effects. The developments have contributed towards the reduction of both the side effects and have also brought about the decreases in frequency and the required dose levels of the therapeutic agents [16]. Photothermal therapy, an emerging method of cancer treatment, utilizes photothermal transduction agents to convert the photoenergy into heat for the thermal ablation of the cancer cells. A previous study has reported Ag_2_S quantum dots with glutathione (GSH-Ag_2_S QDs) as ligands are capable to act as an ideal probe to monitor the therapy, as well as simultaneously exert its therapeutic effects. The HeLa cells were found effectively ablated when the cells were incubated with GSH-Ag_2_S QDs underexposure to 808 nm LASER (light amplification by stimulated emission of radiation) for 5 minutes of duration [17]. Recently, photodynamic therapy (PDT) using ultraviolet (UV) activated photosensitizers have emerged as a potentially effective protocol for treating tumors owing to their high absorbance ability of the experimental UV irradiations [18]. Based on the concept of PDT cancer treatment, titanium dioxide (TiO_2_) NPs have recently been under extensive development as a photosensitizer for cancer cells. This is due to their capability of generating oxidative radicals upon UV irradiations. The TiO_2_ NPs exert the advantages of nontoxicity to biosystems, ease of preparation, as well as high stability in the biological systems [19, 20]. Nonetheless, the magnetic NPs are also under development, and increasing interest concerning their multiple functions including MRI protocols [21], photo-thermal therapy, and targeted drugs and gene deliveries, as well as magnetic enrichments and materials' purification protocols, has been achieved. Additionally, magnetic NPs have also been utilized as a base for preparing core-shell-type nanostructures [22]. This has provided single nanocomposite materials with the capability to perform multiple functions, i.e., therapy, delivery, and bioimagings. The iron oxide (Fe_3_O_4_) NPs (IONPs) properties, also magnetic in nature, have provided several benefits as part of various applications in biomedical fields. This has also included their theranostics applications. IONPs, being the central-core material, are available as part of the applications in delivery module, for conjugation of molecular identification tag, as thermal ablation agent, and as diagnostic imaging probes [23]. The magnetic properties of these nanoparticles and their modifications have also led these materials to selectively accumulate at the tumor site through externally directed magnetic force. Thus, the delivery is considered “targeted” [24]. However, the easy agglomeration of the IONPs has curtailed their utility, and several frontline applications and biomedical approaches of the IONPs have been hindered. Hence, it was deemed pertinent to perform surface functionalization of these nanomaterials through the surface coating and tags conjugation. The making of the core-shell iron oxide-titania NPs by TiO_2_ insertion as the core of the core-shell through following an independent synthetic approach has provided an option in finding metal-based site-specificity to the tumor location, especially the biosystems deep-located and embedded cancers. The core-shell nanocomposite structures are known to increase the composite NPs stability and provide enhanced dispensability, together with magnetically driven delivery and heat generation at the site [24, 25]. The characteristics and requirements have placed the core-shell materials as a potential target for further investigations. However, currently, limited information is available on the potential effects of the nanocomposites prepared by the LASER ablation method. Studies reporting antimicrobial and anticancer activities of the LASER ablation-prepared metal composites and core-shell types NPs are also limited. Therefore, the fabrication of nanocomposites through LASER ablation in a liquid medium without using a catalyst, in the presence and absence of magnetic fields, is a striking option since few reports are available on this aspect of the NPs preparation. The current report aimed to synthesize the composite NPs for use as antimicrobial and antilung cancer agents.

## 2. Materials and Methods

### 2.1. Materials

As target materials, the iron oxide and titania (Fe_3_O_4_, and TiO_2_), both of 99 % purity (Merck, Kondapur, India), were made into pellets, each with a diameter of 9 mm, and utilized to synthesize the iron oxide and titania-based NPs. The ablation process was performed at RT (room temperature) in deionized (DI) water. Dimethyl sulfoxide (DMSO), fetal bovine serum, 3-(4,5- dimethylthiazal-z-yl)-2,5-diphenyltetrazolium (MTT), and doxorubicin were purchased from Sigma Chemical Co., St. Louis, USA. Other used materials included RPMI (Roswell Park Memorial Institute) 1640 (Euro Clone, Milan, Italy) and penicillin and streptomycin (Biosource International, Nivelles, Belgium). All other chemicals and reagents were of analytical grade. Human normal hepatocyte-like WRL-68 cells and human lung adenocarcinoma A549 cell lines were provided by the American Type Culture Collection (ATCC, Manassas, USA).

### 2.2. Microorganisms

The antimicrobial efficacy of the prepared NPs were tested against the clinical isolates of *Escherichia coli* (*E*. *coli*) as Gram-negative and *Staphylococcus aureus* (*S*. *aureus*) as Gram-positive, isolated from the urinary tract and wound infections, respectively. Processing and identification of these isolates were achieved by following the standard biochemical methods at the laboratory. After the transfer of the stock cultures into Mueller–Hinton agar medium, overnight incubation was done at 37°C and stored at 4 °C [26].

Maintenance of the WRL-68 and A549 cell lines were achieved in a mixture of RPMI-1640 and HEPES (20 mM) media, with the latter being used for buffering. Besides, the FCS (5%), sodium pyruvate (10 mM), L-glutamine (2 mM), and either penicillin and/or streptomycin (100 IU mL^−1^) were added. The cells were weekly passaged and retained in the logarithmic growth phase by maintaining the culture in the tissue culture flasks (T 25 cm^2^; Falcon, USA) under a humid atmosphere and optimal conditions (37°C, 5% CO_2_). Afterward, MTT cytotoxicity tests, high-content screening, and cell cycle using a flow cytometer were performed. In parallel, WRL-68 cells were similarly processed for cytotoxicity testing on normal cells [27].

### 2.3. Synthesis of NPs

The synthesis was achieved through the application of LASER ablation in DI water; first, iron oxide pellets were generated by the compression of Fe_3_O_4_ powder and the binder organic material under a hydraulic compressor, followed by sintering at 1000 °C. Nd:YAG LASER (light amplification by stimulated emission of radiation) of 1064 nm wavelength with a pulse duration of 7 ns (nanoseconds) was employed to irradiate the iron oxide target (Figure 1).

The target was fixed at the bottom of a plastic beaker, where the height of the water level over the target was 1 cm, and its volume was 3 milliliters. The LASER values of the fluence utilized for ablation were 30 mJ/cm^2^ and 60 mJ/cm^2^, while the ablation time was 30 min. The second step for the fabrication of the NPs was the same as the steps followed for producing the iron oxide NPs by LASER ablation in liquid. However, in this part, the target material was replaced with titanium oxide, using a liquid that contained iron oxide NPs. All the production steps for the NPs were repeated but under the influence of an external magnetic field with a magnetic fields strength of 0.5 T, as and when applied.

### 2.4. Characterization of the NPs

To characterize the surface morphology and structures of the magnetic field and nonmagnetic fields' presence-synthesized NPs, the transmission electron microscope (TEM, JEM-1200EX, Tokyo, Japan) at an acceleration voltage of 80 kV, and field emission scanning electron microscope (FESEM, JSM-IT800) were used. Size distribution of the particles was obtained on a Malvern Zetasizer Nano ZS90 instrument (Malvern, UK). For the determination of the chemical composition of the NPs, energy dispersive X-ray (EDX) was used, while measurements of the optical absorption were achieved by using a double-beam UV-Vis spectrophotometer (Metertech®, SP8001 spectrophotometer, Japan). The structures and the vibration modes of the NPs were examined by XRD (Philips® PW, Japan) and Raman spectroscopy (Senterra®, Bruker Optics Inc, USA), respectively. A vibration sample magnetometer (VSM) was used to estimate the magnetic saturation and hysteresis loops of the NPs.

### 2.5. Antibacterial Activity of the NPs

The well-diffusion method was applied to examine the activity of the NPs toward the *E*. *coli* and *S*. *aureus*. In brief, separation of the bacteria were achieved at the surface of Mueller–Hinton agar media with about 6 mm diameter wells made by micropipette tip, into which the NPs suspensions with 400 *µ*g mL^−1^ at 30 mJ/cm^2^ and 60 mJ/cm^2^ of the NPs synthesized without and with the presence of magnetic fields were, respectively, used. After incubation for 24 hr, the diameters of the inhibition zones of the nanoparticles-treated plates were measured from various directions with the use of a ruler [28, 29].

### 2.6. Cytotoxic Activity against Cancer Cells

Cancer cell line suspension (200 *μ*L) was seeded at a density of 1 × 10^5^ cells mL^−1^, and prepared in culture plates (96 wells, flat-bottom; Falcon, USA). The cells were then maintained for 48 hrs in the exponential growth phase, treated with concentrations of NPs for 24 hrs, which were as 100, 200, 300, and 400 *µ*g mL^−1^ at 30 mJ/cm^2^ and 60 mJ/cm^2^ of the NPs synthesized without and with the presence of the magnetic fields, respectively, and were labeled with MTT in PBS (100 *µ*L; 10–15 min; 37 °C). The extra stain was discarded and washed with tap water, followed by dissipating the air bubbles in DMSO (50 *µ*L; 10 min). Cell cultures were mounted on a microplate reader (ELx 800, Bio-Tek Instruments Inc., USA), and absorbance was measured at 492 nm [30]. The inhibition percentage was extracted by the following equation:

(1) $$\begin{array}{c} \text{inhibition rate}\left(\%\right)\;=\;\left(Abc-\frac{Abs}{Abc}\right)\times 100, \end{array}$$

where Abc and Abs stands for the values of the control and the tested samples, respectively.

### 2.7. High-Content Screening (HCS) Assay

To further confirm the cytotoxic effects of the synthesized NPs against A549 cells, several related parameters (cell viability, membrane permeability, nuclear intensity, and cytochrome-C) were analyzed using the high-content screening (HCS) assay. A549 cells (1 × 10^5^ density) were seeded in twelve-well plates and incubated (37 °C, 5 % CO_2_, 24 hrs), followed by treatment with various concentrations of magnetic field presence-synthesized NPs. Comparisons were made with untreated and doxorubicin-treated cells (negative and positive controls, respectively). Following an additional 24 hr incubation, cells were treated with a membrane-permeable dye, MMP (excitation 552 nm/emission 576 nm), and cell permeability dye (excitation 491 nm/emission 509 nm) for 1 hr, fixed with 4 % formaldehyde for 15 min, and permeated with 0.1% Triton X-100 in PBS. The reactions were blocked with 3 % bovine serum albumin; afterwards, the cells were incubated with cytochrome-C primary mouse antibody for 1 hr, and cells were washed thrice with wash buffer I (PBS), followed by the addition of DyLight TM 649-conjugated goat antimouse secondary antibodies. Cells were then rinsed with wash buffer II (PBS with 1% Tween-20) before applying Hoechst 33,258 for nuclei staining. The preparations were visualized by using a Cellomics ArrayScan HCS reader (Thermo Scientific, USA). Dye fluorescence intensity was measured through the application of the cell health profiling bioapplication module [31].

### 2.8. Cell Cycle Examinations

A slightly modified method was adopted to analyze the cell cycle [27, 31]. In brief, overnight-seeded A549 cells in a 25 cm^2^ flask, with a concentration of 1 × 10^5^ cell ml ^−1^, were subjected to various concentrations of 24 hr external magnetic field-synthesized NPs (100, 200, and 400 *µ*g mL^−1^). The preparations were fixed with 70% ethanol overnight, then washed twice with PBS, and stained by Cycle TEST TM PLUS DNA Reagent Kit (BD Biosciences, USA) according to the manufacturer's protocol. Cell cycle DNA distribution profile was characterized by flow cytometry (BD Biosciences, USA) for a minimum of 20,000 cells/sample. Percentages of cells passing the cell cycle phases of G1, S, and G2/M were determined by applying Diva software (BD Biosciences, USA).

### 2.9. Statistical Analysis

Significant variances among groups were determined through the use of one-way analysis of variance (ANOVA, Tukey test), where differences were considered as statistically significant at a probability of *P* ≤ 0.05, as determined by using GraphPad Prism software, version 6 (GraphPad Software Inc., La Jolla, CA, USA). Data were expressed in terms of mean ± standard deviation (SD) [32, 33].

## 3. Results and Discussion

### 3.1. Characterization of the NPs

Structures of the NPs were determined by UV-visible absorption spectrum, XRD patterns, TEM, and EDX analyses, followed by FE-SEM. The XRD pattern of the NPs displayed the characteristics diffraction patterns (Figure 2(a)). The XRD peaks recorded at 2*θ* were 28.3°, 33.4°, 40°, 54.4°, and 62.5° which were assigned to the (220), (311), (400), (422), and (440) planes of magnetic Fe_3_O_4_, respectively [34], whereas the peaks observed at 27.4°, 31.6°, 40.9°, 54.3°, 56.5°, and 65.7° were attributed to the (110), (011), (004), (105), (116), and (116) of the TiO_2_ planes, respectively, for these separate, and singular compounds [35].

The XRD patterns of the magnetic and nonmagnetic fields' presence synthesized NPs samples at 30 mJ/cm^2^ and 60 mJ/cm^2^ of LASER fluence energy were determined (Figure 2). Eleven peaks were observed among all the samples which belonged to TiO_2_, Fe_3_O_4,_ and Fe_2_O_3_; four peaks were located at 2*θ* = 20.1°, 25.8°, 27.4°, and 40.3°, corresponding to (100), (110), (100), and (122) planes, respectively, which belonged to the rutile, panguite, and anatase of the TiO_2_ [27]; the three Fe_2_O_3_ peaks were located at 2*θ* of 16.7°, 21.9°, and 56.4°, corresponding to (004), (200), and (105) planes, respectively, belonging to the iron oxide II Fe_2_O_3_, according to JCPDs# 653107 [36]. The four peaks for magnate iron oxide III, Fe_3_O_4_, that were located at 2*θ* of 28.4°, 43.3°, 54.7°, and 64.3°, corresponded to (022), (004), (224), and (044) planes, respectively [34]. On the other hand, the XRD peaks located at 2*θ* of 31.7°, 35.6°, and 47.3°, corresponded to (102), (113), and (133) planes, respectively, were assigned to the sparsely distributed, composite TiFe_2_O_5_ phases [37–39]. The NPs samples showed the corresponding peaks for their constituent metal-oxide presence and also confirmed the presence of the composite nanoparticle materials in the sample, which was mix of different monometallic NPs.  Figure 3 showed the FE-SEM images of the NPs synthesized under magnetic fields and nonmagnetic fields' presence (Figure 4).

Formation of agglomerated and non-agglomerated NPs were observed. The agglomeration was attributed to the magnetic behavior of the iron oxide, Fe_3_O_4_ [40]. Also, the interaction between the plasma plume and the synthesized nanoparticles is plausible in nature. The plume-nanoparticles interaction depends on all attractive and repulsive forces between the plume species, and the NPs, e.g., attractive van der Waals forces, that causes growth through agglomerations. It is plausible that the applications of the magnetic fields during the ablation process caused the changes in the morphology from NPs to berry-like clusters, while the agglomerations led to size increments of the NPs. Applying the magnetic fields during LASER ablation might affect the morphology of the NPs through drifting of the charged, ablated particles (ions and electrons) according to the direction of the magnetic fields' lines. The morphology depends on the mass of the particle, the angle between the LASER plume, and the magnetic field lines angle according to Lorentz's force at plane.

The SEM image revealed the presence of spherical with some core-shell-based NPs [41] which were sparsely distributed. The changes in the morphology were probably due to the changes in the movements of the magnetic core of NPs (Fe_3_O_4_ NPs), which formed parts of some of the NPs structures following the application of the magnetic fields throughout the LASER ablation process [42].

The appearance of Fe, Ti, and O atoms in the EDX spectrum once again demonstrated the composition of the NPs. The results of EDX analysis of the four samples prepared with 30 mJ/cm^2^ and 60 mJ/cm^2^ LASER fluence with the presence and absence of an external magnetic field confirmed this. The percent values of Fe, Ti, and O elements in the NPs prepared in the absence of a magnetic field with a LASER fluence of 30 mJ/cm^2^ were 13.21, 1.61, and 85.18%, respectively. The percentages of Fe, Ti and, O elements in the sample prepared with 60 mJ/cm^2^ were found to be 12.37, 1.67, and 85.96 %, respectively, as shown in the Figures 5(b)–5(d), which exhibited the EDX results of the samples synthesized in the presence and absence of the magnetic fields. The percentages of Fe, Ti, and O atoms in the sample prepared with 30 mJ/cm^2^ LASER fluence were 18.29, 1.7, and 80 %, respectively, while those values for the sample prepared with 60 mJ/cm^2^ LASER fluence were 11.88, 2.36, and 85.67 %, respectively, and confirmed the composite nature of the predominant NPs.

The size and shape of the NPs were determined by TEM (Figure 5). The synthesized nanoparticles were found to be spherical with an average size of ∼70 nm. Since the TiO_2_ shell boundary was clear for some of the NPs, it was easy to visualize in the TEM image. Control of the thickness of the shell layer (i.e., TiO_2_ part) was attempted by using two different energies of the LASER (30 and 60 mJ/cm^2^). This implied that greater energy ablated more material from the target, which precipitated and covered the core material to produce the core-shell material, though this was in lesser ratio. The thickness of the shell was also affected by the presence of a magnetic field which increased the shell layer and led to an increase in the size of some of the NPs [43]. The TEM images also showed the presence of NPs and nanorods with different sizes in the samples prepared under the influence of the magnetic fields. The formation of nanorods can be ascribed to the confinement of plasma that was formed from applying the magnetic fields during the ablation process.

The particle size distributions of the prepared NPs at different conditions were estimated from the dispersion light scattering (DLS) measurements. The LASER fluence and applying of the magnetic fields affected the average particle sizes, agglomeration, and their size distributions. The hydrodynamic diameters of the smallest NPs prepared with 30 mJ/cm^2^ without and with the presence of magnetic fields were 15 nm and 10 nm, respectively. The hydrodynamic diameters of the NPs prepared with 60 mJ/cm^2^ without and with the presence of magnetic fields were ∼20 and 40 nm, respectively.

The energy absorption patterns (Figure 6) of the colloidal NPs samples produced in the presence and absence of an external magnetic fields were recorded. As noticed, the absorption decreased following the application of the magnetic fields, which is possibly due to the increase in the size of the NPs. Increasing the LASER fluence led to an increase in the optical absorbance, also due to an increase in the concentrations of the NPs. An absorption peak was observed at 250 nm for the samples prepared without the presence of the magnetic fields treatment. Another peak was located at 260 nm (Figure 6(b)) which can be assigned to the quantum size effects.

The absorption of the prepared NPs decreased after a wavelength of 200 nm and tended to stabilize after 370 nm. The direct optical energy gap of the NPs were measured by plotting (*αhν*) ^2^ (where *α* is the absorption coefficient and the *hν* is the photon energy) against the photon energy status. The intersection of the linear part (second region) to the photon energy axis generated the energy gap [44, 45], as according to the Tauc plot. As seen (Figure 7(a)), the energy gap values of the nonmagnetic field synthesized NPs with a LASER fluence of 30 mJ/cm^2^ and 60 mJ/cm^2^ were 3.8 and 3.3 eV, respectively, while those of the magnetic field presence synthesized NPs were at 3 eV and 3.5 eV, respectively (Figure 7(b)). This difference can be attributed to the differences in the particle sizes [46].

The indirect energy gap of the NPs were also calculated from (*αhν*) ^0.5^*versus* the photon energy plot. The calculations revealed that the values of 2.4 eV and 2.6 eV in the absence of an external magnetic field (Figure 8(a)) and 1.5 eV and 1.2 eV values, under the effects of the presence of an external magnetic fields for samples prepared with 30 mJ/cm^2^ and 60 mJ/cm^2^, respectively, were observed (Figure 8(b)).

Raman spectra, of the magnetic fields and nonmagnetic field's presence of the synthesized and major constituent NPs, are shown in Figure 9. The results showed that the vibration modes were centered at 91 cm^−1^ (*E*_g_), 144 cm^−1^ (*E*_g_), 396 cm^−1^ (B_1g_), 512 cm^−1^ (B_1g_), 541 cm^−1^ (B_1g_ + *A*_1g_), and 609 cm^−1^ (*E*_g_).

These modes were assigned to anatase and rutile phases semblances of the TiO_2_, which is consistent with the XRD results. The three vibration modes were assigned, based on semblances, to the magnetite, Fe_3_O_4_, and were observed at 145^−1^ (T_2g_), 302 cm^−1^ (T_2g_), and 554 cm^−1^ (T_1g_). On the other hand, five peaks observed at 225 cm^−1^ (A_1g_), 254 cm^−1^ (*E*_g_), 355 cm^−1^ (*E*_g_), 444(A_1g_) cm^−1^, and 604 cm^−1^ (*E*_g_) were allotted to the iron oxide II, Fe_2_O_3_ phase, based on the peaks patterns and reported data. These results were consistent with those reported by Benjwal [47], Verma[48], and Salim *et al.* [49].  Figure 10 showed the magnetization plot of the NPs. An affirmed superparamagnetic behavior was observed, which suggested potential applications of these NPs in optoelectronics and biomedicine, among others applications [50]. The VSM results showed that the NPs prepared in presence of the magnetic fields exhibited a narrow hysteresis loop with coercivity (Hc) of 1.67 Oe, while the NPs prepared at B0 have Hc of 10.35 Oe, thereby indicating that the NPs prepared in the presence of magnetic field have superparamagnetic behavior.

### 3.2. Antibacterial Activity of the NPs

Images shown in Figure 11 demonstrated the antibacterial effects, of the magnetic fields and nonmagnetic field's presence of the synthesized NPs, as indicated by the diameters of the inhibition zones. *S*. *aureus* responded with an inhibition zone of a larger diameter as compared to that of the *E*. *coli* under similar concentrations and conditions. The activity of the NPs synthesized with the magnetic fields' presence showed 28.00 ± 1.46 mm and 30.76 ± 1.24 mm zones of inhibition for the *E*. *coli*; 28.76 ± 1.42 mm and 31.23 ± 2.46 mm of inhibition zones for the *S*. *aureus*, which was stronger than that recorded for the NPs synthesized without the presence of magnetic field (24.76 ± 1.50 mm and 25.66 ± 2.22 mm zones of inhibitions for *E*. *coli*; 26.00 ± 2.40 mm and 27.66 ± 2.20 mm zones of inhibitions for the *S*. *aureus*). These outcomes suggested higher sensitivity of the *S*. *aureus* to the magnetic-field-present synthesized NPs as compared to that of the *E*. *coli*. The NPs exerted typical characteristics of antibacterial effect against both the Gram-negative and Gram-positive bacteria, which were also demonstrated by the activity of the NPs against the growth of *S*. *aureus*[51–53]. The activity of the both types, of magnetic fields and nonmagnetic fields presence synthesized, NPs suggested the possibility of the presence of variable antibacterial pathways against *E*. *coli* and *S*. *aureus*. For Gram-negative bacteria, the resistance is considered to be mainly conferred by the transporters that are situated within the membrane. These transporters, known as multidrug efflux pumps, confer protection to the bacterial cells against the action of antibiotic agents on both sides of the membrane [54]. The study of Wu et al. demonstrated that the Ag NPs (silver nanoparticles) exhibit antibacterial properties, and their potentials were increased with the decreasing particles sizes. The antibacterial activities were also attributed to the contact action of Ag NPs with microbes, and the released silver ions which have strong bonding abilities with functional groups of cellular contents were playing the part. The mechanism of cell death suggested that the NPs are adsorbed on the cytoderm of bacterial entities, and they penetrate the cytomembrane to disturb the normal functions of the cells, which results in apoptosis [55]. Moreover, it was also found out that silver nanoparticles-decorated hydroxyapatite (HA@Ag) nanocomposites were having excellent properties of inhibiting and killing the bacteria, which were especially prominent for the Gram-positive bacteria, *S*. *aureus*, and that were better than the used HA NPs, and the Ag NPs alone [56].

Another earlier study revealed that the cell bodies of the *E*. *coli* were easily susceptible to distortion and rupture in response to the reactive incoming species. Nevertheless, in the case of *S*. *aureus*, the membrane destruction was not observed, while cell surfaces were massively covered by the presence of NPs. This interaction seemed to cause restriction in the bacterial activities and may have disturbed the functions of the selectively permeable barriers that eventually lead to the cells death [57]. Researches that have particularly focused on antimicrobial mechanisms have provided evidence of inactivation of the bacterial cells at the levels of regulatory networks and the signaling in bacteria, for the bacteria, which were treated with photocatalytic NPs. These effects were associated with remarkably reduced respiratory chain activity and inhibited the capability of assimilating and transporting iron and phosphorous. Such mechanisms, along with the extensively altered cell wall and cell membranes, were considered as the principal and plausible explanations for the biocidal activity of the NPs [58]. Results of the present study suggested that the presence of magnetic field-produced NPs caused a slightly enhanced bacterial cells death. However, another earlier study reported the largest inhibition zones in both the *S*. *aureus* and *E*. *coli*, with more potent effects for the TiO_2_ NPs, prepared under the magnetic field's presence, when compared with the NPs prepared without the presence of a magnetic field [59].

### 3.3. MTT Assays

Figure 12 demonstrated the viability of A549 cells in response to treatment with four concentrations of the magnetic fields and non-magnetic field's presence synthesized NPs. The treatment with NPs synthesized under the influence of magnetic fields resulted in significantly reduced viability (*P* ≤ 0.05). This inhibition was higher than that observed in response to NPs synthesized without the presence of an external magnetic field. The effects were also concentration-dependent. The inhibitory concentration (IC_50_) values of A549 cells at 30 mJ/cm^2^ and 60 mJ/cm^2^ of the NPs synthesized under the presence of the magnetic field was 190 *μ*g mL^−1^ and 165 *μ*g mL^−1^.

The inhibition trends exerted by the NPs synthesized without the presence of magnetic fields at 60 mJ/cm^2^ revealed cytotoxicity values of 43.2 %, 40.0 %, 58.2 %, and 58.8 %, respectively, whereas the higher cytotoxicity values were observed at a concentration of 400 *μ*g mL^−1^. The NPs synthesized under the presence of the magnetic fields, at the same LASER pulse energies, showed the strongest activity, which was significantly higher than that observed for the other treatments. On the contrary, the normal cell lines responded with slight cytotoxicity to treatments. For all the conditions, the cell viability values at 400 µg ml^−1^ were 80.0 %, 90.0 %, 80.0 %, and 79.6 %, respectively (Figures 12(a)–12(d)).

The proposed mechanisms of the anticancer activity of these NPs can be explained by the ability of NPs to generate ROS (Reactive Oxygen Species), even in absence of light that can cause changes in biomacromolecules, such as, proteins, nuclei acids, and lipids in response to the effects of the generated oxidative stress in the cells and tissues. These oxygen species produce free radicals that are short-lived and unstable, and which influence the nuclear viability and healthiness conditions of the affected organisms, and finally leads to cells death. The ROS also cause oxidation of proteins and peroxidation of lipids that leads to damaging the fluidity of the cell membrane, thereby changing the permeability of fluids and ion transports across it, and cause inhibition of metabolic processes [30]. The mechanism describing the cytotoxicity caused to the malignant cells by magnetic NPs was first proposed by Gupta and Gupta. In this mechanism, the surfactants of the NPs were supposed to interact with the proteins on the surface of the cancer cell through an -NH_2_ (amine) functional group bindings. The magnetic NPs have the tendency of aggregation and, subsequently, adsorbed on the plasma proteins surfaces and in the protein grooves. Following their entry into the cells, the NPs show tendency of forming necklace-like eccentric circles around the nucleus, and as a consequence, the endocytosis causes the formation of cell bubbles, followed by induction of cell death through apoptosis [60].

The cellular mechanism of NPs affected cell death and apoptosis is still under investigation for differently conditioned and various kinds of NPs. The synergistic and augmenting roles of different metal-based magnetic and non-magnetic NPs are also being continuously getting attention for their various anticancer activities. Nonetheless, the present findings suggested that the NPs may have the possibility of augmenting the cytotoxic effects of the drugs, in addition to its own anticancer properties, and it can also be used as part of the combined chemotherapy. Also, the potential of these NPs can be further developed for combined sonodynamic chemotherapy for viable cancers.

### 3.4. High-Content Screening (HCS) Assay of A549

The cytotoxic activities of the NPs synthesized with the presence of the magnetic fields at 60 mJ/cm^2^ were determined by using an HCS assay. The alterations in the A549 cell lines which were detected based on several parameters, including nuclear intensity, membrane permeability, MMP, and cytochrome-C conditions. For comparison purposes, the doxorubicin was employed as a positive control, whereas untreated cells served as another control (negative control). Images of the A549 cells following treatments with tested concentrations of the NPs, as well as those of the controls, were compared through Figures 13 and 14.

### 3.5. Total Nuclear Intensity

The exposure of A549 cell lines to the NPs caused an increase in the size of the nuclei that might have resulted from the swellings. This influence was shown to be concentration-dependent. Following their staining with Hoechst blue, the nuclei appeared mostly condensed as a result of exposure to the NPs at 400 *µ*g mL^−1^ (1-fold increase in the nuclear fluorescence intensity). These differences were shown to be significant (*P* < 0.01) in comparison with the untreated cells. No similar influences were observed in response to treatment with 25–50 *µ*g mL^−1^ (data not presented). However, the treatment with the positive control, doxorubicin, resulted in a 1.2-folds increase in the nuclear intensity. The nuclei appeared condensed with bright intensity. Cells also demonstrated typical characteristics of the observable morphology of the apoptotic cells. These included the condensations and fragmentations of the nuclei, shrinkage of the cells, production and aggregation of apoptotic bodies [61]. This type of treatment could have possibly activated an altered mitochondrial function, which might have caused the cell death either by necrosis, or apoptosis. These events possibly led to the loss of membrane potential of the mitochondria, followed by the release of cytochrome-C.

### 3.6. Cellular Membrane Permeability

As shown in Figure 14, the permeability of the cell membranes in A549 cells were altered in response to the exposure to two concentrations of the NPs. A significant increase (*P* < 0.01) of 0.5 and 1.2 folds were observed in the cells treated with 200 *µ*g mL^−1^ and 400 *µ*g mL^−1^ concentrations of the NPs synthesized under the presence of magnetic fields at 60 mJ/cm2 LASER fluence, respectively, in comparison with the control cells (Figure 14). Nonetheless, the treatment with doxorubicin resulted in an increase of 2.4-folds in the permeability of cell membranes. These findings confirmed the induction of apoptosis in malignant cells in response to the NPs, which was evident through the increase in the permeability of the dye. The cell membrane permeability is commonly correlated to toxic and/or apoptotic reactions. Any distortion in cell membrane integrity is considered a typical phenotypic characteristic of the obvious cytotoxicity [62]. Such reactions are typically observed upon the loss of plasma membrane integrity. Consequently, a variety of cell death pathways act on the induction of particular reshuffling events within the membrane [63]. The NPs altered both the structure and organization of the intracellular and membrane-associated lipid layers to cause these effects. The events are also capable of altering the membrane permeability in response to a second messenger mechanism, such as that of the phospholipase pathway which is associated with the continuous activation of the protein kinase C, thereby eventually leading to cell lysis [64].

### 3.7. Mitochondrial Membrane Potential (MPP)

To better characterize the signaling pathways leading to cell death during the exposure of A549 cells to the toxic agents, the influences of the NPs, synthesized under the presence of magnetic fields at 60 mJ/cm^2^ LASER fluence, were examined on the membrane permeability of the mitochondria. For this purpose, MMP dye was applied and analyzed. A significant decrease (20%, *P* < 0.01), following treatment with a concentration of 200 *µ*g mL^−1^of the NPs was observed. The treatment with 400 *µ*g mL^−1^ caused a reduction of 35% as compared to the positive control which revealed a decrease of 70%, as compared to the untreated cells. The mean intensity of the MMP that penetrated the mitochondrial membrane was the basis of MPP determination, and a lower fluorescent intensity reflected a stronger impact on the mitochondria. Apoptosis, a mechanism, which has essential contributions to the activities of development, differentiation, and homeostasis, was thus confirmed. During the course of cancer development, dysregulation of the apoptosis process is commonly observed. In most cases, proper apoptosis is triggered through the event of mitochondrial outer membrane permeability (MOMP). This characterizes the mitochondrial (intrinsic) pathway and ultimately leads to activation of the caspase pathway and cleavage of the protein substrate [65].

### 3.8. Cytochrome-C Release

The findings of the study revealed weak and diffused staining of the cytochrome-C within the cells of the control sample. On the contrary, A549 cells exposed to treatments with the 200 µg mL^−1^ and 400 µg mL^−1^ of NPs synthesized under the presence of magnetic fields at 60 mJ/cm^2^ LASER fluence, as well as those treated with doxorubicin, demonstrated strong staining patterns around their nuclei (Figure 14). The release of cytochrome-C showed an increase of 1.2, 1.6, and 2.0-folds of fluorescent intensity, compared to the untreated cells. These results suggested a higher translocation of the cytochrome-C from the mitochondrial site to the cytosol in response to the treatments with the NPs. Sporadically, cytochrome-C was also observed inside the nuclei of the treated cells, but not in the control cells. Upon its release, the cytochrome-C activates a cascade of caspases and cysteine proteases, the major players in cellular degradation and self-digestion. The cytochrome-C is known for its major role in apoptosis, and when its release from the mitochondria to the cytoplasm is observed, it leads to the activation of the caspase pathway, and therefore the cell's commitment to the apoptotic pathway is established. Accordingly, the release of cytochrome-C was proposed to be a consequence of the mitochondrial matrix swelling, which is, in turn, triggered by the apoptotic stimuli [66].

### 3.9. Cell Cycle Distributions

Figure 15 demonstrated the results of cell-cycle distribution which were obtained by flow cytometry, as determined through the percentages of G1, S, and G2/M cell populations. A significant increase (*P* ≤ 0.05) was recorded in the percentages of G1 phase cells (58.88%, 60.20%, and 66.90%) in response to the treatments with the NPs synthesized under the presence of magnetic fields at 60 mJ/cm^2^ LASER fluence, at 100 *µ*g mL^−1^, 200 *µ*g mL^−1^, and 400 *µ*g mL^−1^, respectively.

However, no significant differences were found concerning the cells in the S phase. The cells in phase G2/M demonstrated significant reductions in their percent values (19.30%, 16.10%, and 12.70%) following the treatments with 100 *µ*g mL^−1^, 200 *µ*g mL^−1^, and 400 *µ*g mL^−1^ concentrations, respectively, of the NPs synthesized under the presence of magnetic fields at 60 mJ/cm2 LASER fluence. Based on these results, it was suggested that the NPs were capable of inducing A549 cell cycle arrest at the G1 phase. Such an influence can be attributed to the enhanced potential of the NPs to penetrate and accumulate within the A549 cells, which consequently boost their cytotoxicity through the generation of ROS. Parallel results were obtained from the magnetic iron NPs on the production of intracellular ROS. As a result, the oxidative stress against human breast cancer (AMJ-13 and MCF-7) and ovarian (SKOV-3) cancer cells were increased. Consequently, the cancer cell nuclei were found condensed, and chromosomal DNA was fragmented, which eventually led to cell death [67–69].

## 4. Conclusion

The iron oxide-titania composite, core-shell, and monometallic NPs were prepared through LASER ablation in a liquid medium without the presence of any catalyst. Also, during the NP preparation, the preparative process was exposed to an external magnetic field. The impacts on the properties of NPs because of the presence of the magnetic fields during synthesis of NPs were investigated. Simultaneous applications of magnetic fields and ablation process resulted in alterations in the morphology of NPs, which culminated in generation of Berry-like clusters in addition to the production of the NPs. The energy gap value of the NPs prepared with the presence of the magnetic fields was higher than the NPs prepared without the presence of any magnetic fields. Based on these results, it was concluded that the NPs prepared under the influence of magnetic fields have significantly greater potentials than those prepared without the presence of the magnetic fields. The NPs also converted from having paramagnetic to superparamagnetic properties after applying the magnetic fields during the LASER ablation process. The results also showed that these NPs exhibit excellent antibacterial properties against both Gram-negative bacteria of *E*. *coli* and Gram-positive bacteria of *S*. *aureus*. The potentials of the magnetic fields were stronger than those recorded for the NPs synthesized without the presence of a magnetic field. Comparatively, higher cytotoxicity levels against lung cells (A549), as compared to the low cytotoxicity against normal cell line (WRL-68), were observed. The treatment with the NPs produced under a magnetic field resulted in significantly reduced viability of the A549 cell lines. This inhibition was higher than that observed in response to the NPs synthesized without the presence of an external magnetic field. These impacts against cancer cells enhanced the cell cycle arrests at the G1 phase. Both, the effectiveness of these NPs as anticancer agents and their particular capability of targeting the breast cancer cells need to be further investigated in more detail for a better understanding of the NPs impacts, especially the NPs prepared under the influence of the presence of a magnetic field. The present study indicated the potential of the synthesized NPs in treating certain microbial infections and cancers in combination with the classical chemotherapy involving synthetic-, recombinant-, and natural products-based drugs need to be evaluated. In addition, based on the obtained results, the synthesized NPs could also be a useful sonosensitizer in sonomagnetic heating and therapy for cancer and other viable conditions of different diseases.

Of lately, preparative report on iron oxide, and iron oxide-titania core-shell nanoparticles of differently-averaged size, and characteristics have also appeared. The photo-reduction properties of the prepared nanoparticles have been studied, which could lead to details in biomechanistic aspects in light-sensitive materials, and may provide a lead for better metal-based photo-sensitive reactions, and probably anti-cancer properties [70, 71].

## Figures and Tables

**Figure 1:** Schematic illustration of NPs production through the LASER ablation procedure in liquid medium.

**Figure 2:** (a) XRD patterns of the NPs prepared by LASER ablation in liquid medium with a LASER fluence of 60 mJ/cm^2^ and (b) XRD patterns of the NPs prepared by LASER ablation in liquid medium with a LASER fluence of 30 mJ/cm^2^ and 60 mJ/cm^2^ without and with the presence of the magnetic fields. The XRD peaks located at 2θ of 31.7°, 35.6°, and 47.3°, corresponding to (102), (113), and (133) planes, were assigned for the TiFe_2_O_5_ phase. M stands for the magnetic field.

**Figure 3:** FE-SEM images of the prepared NPs: without applying a magnetic field and the LASER fluence: (a) 30 mJ/cm^2^ and (b) 60 mJ/cm^2^; with applying a magnetic field and the LASER fluence: (c) 30 mJ/cm^2^ and (d) 60 mJ/cm^2^.

**Figure 4:** EDX of the NPs prepared: without applying a magnetic field and the LASER fluence: (a) 30 mJ/cm^2^ and (b) 60 mJ/cm^2^; with applying a magnetic field and the LASER fluence: (c) 30 mJ/cm^2^ and (d) 60 mJ/cm^2^.

**Figure 5:** TEM images of the NPs prepared: without applying a magnetic field and the LASER fluence: (a) 30 mJ/cm^2^ and (b) 60 mJ/cm^2^; with applying a magnetic field and the LASER fluence: (c) 30 mJ/cm^2^ and (d) 60 mJ/cm^2^.

**Figure 6:** The optical absorbance of the NPs, prepared by LASER ablation in liquid medium with a LASER fluence of 30 mJ/cm^2^ and 60 mJ/cm^2^: (a) without the presence of the magnetic field and (b) with the presence of the magnetic field.

**Figure 7:** The (*α*h*ν*) ^2^*versus* photon energy plot of the NPs prepared by LASER ablation in liquid medium with a LASER fluence of 30 mJ/cm^2^ and 60 mJ/cm^2^: (a) without the presence of the magnetic field and (b) with the presence of the magnetic field.

**Figure 8:** The (*α*h*ν*) ^0.5^*versus* photon energy plot of the NPs prepared by LASER ablation in liquid with a LASER fluence of 30 and 60 mJ/cm^2^: (a) without the magnetic field and (b) with the presence of the magnetic field.

**Figure 9:** Raman spectra of the major constituent NPs.

**Figure 10:** Magnetization activity of the synthesized NPs measured with VSM. (a) VSM without external magnetic field and (b) VSM with external magnetic field. (c) The photograph shows the effects of external magnetic field on the NPs.

**Figure 11:** Antibacterial activity of the synthesized NPs against *E*. *coli* (blue-lined graph) and *S*. *aureus* (red-lined graph). A, control bacterial strain without treatment; B and C, 30 mJ/cm^2^ and 60 mJ/cm^2^ of the NPs synthesized without the presence of magnetic field; and D and E with the presence of magnetic fields, respectively. ^*∗∗∗∗*^*P* ≤ 0.0001.

**Figure 12:** Antiproliferative activity of the NPs against A549 and WRL68 cells. (a, b) Cells were treated with the NPs synthesized by 30 mJ/cm^2^ and 60 mJ/cm^2^ without magnetic field, respectively. (c, d) Cells were treated with the NPs synthesized by 30 mJ/cm^2^ and 60 mJ/cm^2^ with the magnetic field, respectively. 100, 200, 300, and 400 *µ*g mL^−1^ were used.

**Figure 13:** Multiparameter cytotoxicity analysis of A549 cells treated with the NPs synthesized under the presence of magnetic field at 60 mJ/cm^2^. Doxorubicin was the positive control (1 mM) at 200 *µ*g mL^−1^, and 400 *µ*g mL^−1^ concentrations.

**Figure 14:** Effects of the NPs synthesized under the presence of magnetic field at 60 mJ/cm^2^ against A549 cells. The effects were assessed using the ArrayScan HCS Reader; ^*∗*^*P* ≤ 0.05; ^*∗∗*^*P* ≤ 0.01.

**Figure 15:** Flow cytometry assessment of cell cycle distribution (G1, (S), and G2/M) of A549 cells treated with different concentrations of the NPs synthesized with the magnetic field at 60 mJ/cm^2^ for 24 hrs. (a) Negative control; (b–d) 100, 200, and 400 *µ*g mL^−1^, respectively; (e) Statistical analysis of cell cycle distribution. ^*∗*^*P* ≤ 0.05; ^*∗∗*^*P* ≤ 0.01.

## Data Availability

No data were used to support this study.

## References

[1] Shen S., Wu L., Liu J. (2015). Core-shell structured Fe3O4@TiO2-doxorubicin nanoparticles for targeted chemo-sonodynamic therapy of cancer. *International Journal of Pharmaceutics*.

[2] Chen Y., Gao Y., Li Y., Wang K., Zhu J. (2019). Synergistic chemo-photodynamic therapy mediated by light-activated ROS-degradable nanocarriers. *Journal of Materials Chemistry B*.

[3] Kharissova O. V., Kharisov B. I., Oliva González C. M., Méndez Y. P., López I. (2019). Greener synthesis of chemical compounds and materials. *Royal Society Open Science*.

[4] Amoabediny G. H., Naderi A., Malakootikhah J. (2009). Guidelines for safe handling, use and disposal of nanoparticles. *Journal of Physics: Conference Series*.

[5] Zahin N., Anwar R., Tewari D., Kabir M. T. (2020). Nanoparticles and its biomedical applications in health and diseases: special focus on drug delivery. *Environmental Science & Pollution Research*.

[6] de Kraker M. E., Stewardson A. J., Harbarth S. (2016). Will 10 million people die a year due to antimicrobial resistance by 2050. *PLoS Medicine*.

[7] Toner E., Adalja A., Gronvall G. K., Cicero A., Inglesby T. V. (2015). Antimicrobial resistance is a global health emergency. *Health Security*.

[8] Song L., Kolar M., Xing E. P. (2009). Keller: estimating time-varying interactions between genes. *Bioinformatics*.

[9] Ito K., Suda T. (2014). Metabolic requirements for the maintenance of self-renewing stem cells. *Nature Reviews Molecular Cell Biology*.

[10] Shen S. P., Aleksic J., Russell S. (2013). Identifying targets of the Sox domain protein Dichaete in the Drosophila CNS via targeted expression of dominant negative proteins. *BMC Developmental Biology*.

[11] El-Dakdouki M. H., Xia J., Zhu D. C. (2014). Assessing the in vivo efficacy of doxorubicin loaded hyaluronan nanoparticles. *ACS Applied Materials & Interfaces*.

[12] Ashikaga T., Wada M., Kobayashi H. (2000). Effect of the photocatalytic activity of TiO2 on plasmid DNA. *Mutation Research: Genetic Toxicology and Environmental Mutagenesis*.

[13] Shkodenko L., Kassirov I., Koshel E. (2020). Metal oxide nanoparticles against bacterial biofilms: perspectives and limitations. *Microorganisms*.

[14] Turner R. J. (2017). Metal-based antimicrobial strategies. *Microbial biotechnology*.

[15] Miller K. D., Nogueira L., Mariotto A. B. (2019). Cancer treatment and survivorship statistics. *CA: A Cancer Journal for Clinicians*.

[16] Senapati S., Mahanta A. K., Kumar S., Maiti P (2018). Controlled drug delivery vehicles for cancer treatment and their performance. *Signal transduction and targeted therapy*.

[17] Gao M., Zhao H., Wang Z. (2021). Controllable preparation of Ag_2_S quantum dots with size-dependent fluorescence and cancer photothermal therapy. *Advanced Powder Technology*.

[18] Zhang H., Shan Y., Dong L. (2014). A comparison of TiO2 and ZnO nanoparticles as photosensitizers in photodynamic therapy for cancer. *Journal of Biomedical Nanotechnology*.

[19] Khan S. T., Ahmad F., Shahadat M., Rehman W. U., Khan A. M. (2020). Metal and metal oxide nanoparticles for water decontamination and purification. *Environmental Nanotechnology for Water Purification*.

[20] Khashan K. S., Sulaiman G. M., Abdulameer F. A. (2021). Antibacterial activity of TiO2 nanoparticles prepared by one-step laser ablation in liquid. *Applied Sciences*.

[21] Sun C., Lee J. S. H., Zhang M. (2008). Magnetic nanoparticles in MR imaging and drug delivery. *Advanced Drug Delivery Reviews*.

[22] Ken K. R., Mariana R., Natasha D., Koiti A. (2021). Titanium and iron oxide nanoparticles for cancer therapy: surface chemistry and biological implications. *Frontiers in Nanotechnology*.

[23] Khashan S., Dagher S., Tit N. (2017). Novel method for synthesis of Fe_3_O_4_@TiO_2_ core/shell nanoparticles. *Surface and Coatings Technology*.

[24] Sunaryono S., Fitriana D. R., Novita L. R. (2020). The effect of Fe3O4 concentration to photocatalytic activity of Fe3O4@TiO2-PVP core-shell nanocomposite. *Journal of Physics: Conference Series*.

[25] Chen H., Zhang L., Li M., Xie G. (2020). Synthesis of core-shell micro/nanoparticles and their tribological application: a Review. *Materials*.

[26] Jabir M. S., Nayef U. M., Jawad K. H., Taqi Z. J., H B. A., Ahmed N. R. (2018). Porous silicon nanoparticles prepared via an improved method: a developing strategy for a successful antimicrobial agent against *Escherichia coli* and *Staphylococcus aureus*. *IOP Conference Series: Materials Science and Engineering*.

[27] Sulaiman G. M. (2016). Molecular structure and antiproliferative effect of galangin in HCT-116 cells: in vitro study. *Food science and biotechnology*.

[28] Jahangirian H., Haron M. J., Shah M. H. (2013). Well diffusion method for evaluation of antibacterial activity of copper phenyl fatty hydroxamate synthesized from canola and palm kernel oils. *Digest Journal Nanomat Biostruc*.

[29] Ismail R. A., Sulaiman G. M., Mohsin M. H., Saadoon A. H. (2018). Preparation of silver iodide nanoparticles using LASER ablation in liquid for antibacterial applications. *IET Nanobiotechnology*.

[30] Khashan K. S., Sulaiman G. M., Hussain S. A., Marzoog T. R., Jabir M. S. (2020). Synthesis, characterization and evaluation of antibacterial, antiparasitic and anticancer activities of aluminum-doped zinc oxide nanoparticles. *Journal of Inorganic and Organometallic Polymers and Materials*.

[31] Al-Dulimi A. G., Al-Saffar A. Z., Sulaiman G. M. (2020). Immobilization of l-asparaginase on gold nanoparticles for novel drug delivery approach as anticancer agent against human breast carcinoma cells. *Journal of Materials Research and Technology*.

[32] Kareem S. H., Naji A. M., Taqi Z. J., Jabir M. S. (2020). Polyvinylpyrrolidone loaded-MnZnFe2O4 magnetic nanocomposites induce apoptosis in cancer cells through mitochondrial damage and P53 pathway. *Journal of Inorganic and Organometallic Polymers and Materials*.

[33] Sulaiman G. M., Ali E. H., Jabbar I. I. (2014). Synthesis, characterization, antibacterial and cytotoxic effects of silver nanoparticles. *Digest Journal Nanomat Biostructure*.

[34] Sasaki S. (1997). Radial distribution of electron density in magnetite, Fe3O4. *Acta Crystallographica Section B Structural Science*.

[35] Kalaiarasi S., Jose M. (2017). Dielectric functionalities of anatase phase titanium dioxide nanocrystals synthesized using water-soluble complexes. *Applied Physics A*.

[36] Karlsson N. (1951). Metallic oxides with the structure of high-speed steel carbide. *Nature*.

[37] Wechsler B. A., Lindsley D. H., Prewitt C. T. (1984). ” Crystal structure and cation distribution in titanomagnetites (Fe_3_-xTixO_4_). *American Mineralogist*.

[38] Harrison R. J., Redfern S. A. T. (2001). Short- and long-range ordering in the ilmenite-hematite solid solution. *Physics and Chemistry of Minerals*.

[39] Obaidat I., Nayek C., Manna K., Bhattacharjee G., Al-Omari I., Gismelseed A. (2017). Investigating exchange bias and coercivity in Fe3O4-*γ*-Fe2O3 core-shell nanoparticles of fixed core diameter and variable shell thicknesses. *Nanomaterials*.

[40] Bursill L. A., Grey I. E., Lloyd D. J. (1976). High-temperature rutile-derived crystallographic shear structures. I. (020)r CS structures. *Journal of Solid State Chemistry*.

[41] Baker C., Ismat Shah S., Hasanain S. K. (2004). Magnetic behavior of iron and iron-oxide nanoparticle/polymer composites. *Journal of Magnetism and Magnetic Materials*.

[42] Farrokhi H., Gruzdev V., Zheng H., Zhou W. (2019). Fundamental mechanisms of nanosecond-LASER-ablation enhancement by an axial magnetic field. *Journal of the Optical Society of America B*.

[43] Song H.-M., Wei Q., Ong Q. K., Wei A. (2010). Plasmon-resonant nanoparticles and nanostars with magnetic cores: synthesis and magnetomotive imaging. *ACS Nano*.

[44] Ismail R. A., Mousa A. M., Khashan K. S. (2016). Synthesis of PbI_2_ nanoparticles by LASER ablation in methanol. *Journal of Materials Science: Materials in Electronics*.

[45] Ismail R. A., Fadhil F. A. (2014). Effect of electric field on the properties of bismuth oxide nanoparticles prepared by LASER ablation in water. *Journal of Materials Science: Materials in Electronics*.

[46] Ismail R. A., Abdulrazaq O. A., Yahya K. Z. (2005). Preparation and characterization of In2o3 thin films for optoelectronic applications. *Surface Review and Letters*.

[47] Benjwal P., Kumar M., Chamoli P., Kar K. K. (2015). Enhanced photocatalytic degradation of methylene blue and adsorption of arsenic(iii) by reduced graphene oxide (rGO)-metal oxide (TiO2/Fe3O4) based nanocomposites. *RSC Advances*.

[48] Verma R., Gangwar J., Srivastava A. K. (2017). Multiphase TiO2nanostructures: a review of efficient synthesis, growth mechanism, probing capabilities, and applications in bio-safety and health. *RSC Advances*.

[49] Salim E. T., Ismail R. A., Halbos H. T. (2019). Growth of Nb2O5 film using hydrothermal method: effect of Nb concentration on physical properties. *Materials Research Express*.

[50] Szatkowski T., Wysokowski M., Lota G. (2015). Novel nanostructured hematite-spongin composite developed using an extreme biomimetic approach. *RSC Advances*.

[51] Ruíz-Baltazar Á. D. J., Méndez-Lozano N., Larrañaga-Ordáz D., Reyes-López S. Y., Zamora Antuñano M. A., Pérez Campos R. (2020). Magnetic nanoparticles of Fe3O4 biosynthesized by cnicus benedictus extract: photocatalytic study of organic dye degradation and antibacterial behavior. *Processes*.

[52] Azam A., Ahmed A. S., Oves M., Khan M. S., Habib S. S., Memic A. (2012). Antimicrobial activity of metal oxide nanoparticles against Gram-positive and Gram-negative bacteria: a comparative study. *International Journal of Nanomedicine*.

[53] Ismail R. A., Sulaiman G. M., Abdulrahman S. A., Marzoog T. R. (2015). Antibacterial activity of magnetic iron oxide nanoparticles synthesized by laser ablation in liquid. *Materials Science and Engineering: C*.

[54] Higgins C. F. (2007). Multiple molecular mechanisms for multidrug resistance transporters. *Nature*.

[55] Wu Y., Yang Y., Zhang Z., Wang Z., Zhao Y., Sun L. (2018). A facile method to prepare size-tunable silver nanoparticles and its antibacterial mechanism. *Advanced Powder Technology*.

[56] Ni Z., Gu X., He Y. (2018). Synthesis of silver nanoparticle-decorated hydroxyapatite (HA@ Ag) poriferous nanocomposites and the study of their antibacterial activities. *RSC Advances*.

[57] Buckley A., Turner J. R. (2018). Cell biology of tight junction barrier regulation and mucosal disease. *Cold Spring Harbor Persp Biol*.

[58] de Dicastillo C. L., Correa M. G., Martínez F. B., Streitt C., Galotto M. J. (2020). Antimicrobial Effect of Titanium Dioxide Nanoparticles. *Antimicrob Resist-A One Health Persp, IntechOpen*.

[59] Bahjat H. H., Ismail R. A., Sulaiman G. M., Jabir M. S. (2021). Magnetic field-assisted LASER ablation of titanium dioxide nanoparticles in water for antibacterial applications. *Journal of Inorganic and Organometallic Polymers and Materials*.

[60] Gupta A. K., Gupta M. (2005). Synthesis and surface engineering of iron oxide nanoparticles for biomedical applications. *Biomaterials*.

[61] Doonan F., Cotter T. G. (2008). Morphological assessment of apoptosis. *Methods*.

[62] Bucciantini M., Calloni G., Chiti F. (2004). Prefibrillar amyloid protein aggregates share common features of cytotoxicity. *Journal of Biological Chemistry*.

[63] Zhang Y., Chen X., Gueydan C., Han J. (2018). Plasma membrane changes during programmed cell deaths. *Cell Research*.

[64] Qiu Z. H., Leslie C. C. (1994). Protein kinase C-dependent and-independent pathways of mitogen-activated protein kinase activation in macrophages by stimuli that activate phospholipase A2. *Journal of Biological Chemistry*.

[65] Redza-Dutordoir M., Averill-Bates D. A. (2016). Activation of apoptosis signaling pathways by reactive oxygen species. *Biochimica et Biophysica Acta (BBA) - Molecular Cell Research*.

[66] Desagher S., Martinou J. C. (2000). Mitochondria as the central control point of apoptosis. *Trends in Cell Biology*.

[67] Sulaiman G. M., Tawfeeq A. T., Naji A. S. (2018). Biosynthesis, characterization of magnetic iron oxide nanoparticles, and evaluations of the cytotoxicity and DNA damage of human breast carcinoma cell lines. *Artif Cells Nanomed Biotech*.

[68] Jabir M. S., Nayef U. M., Abdulkadhim W. K. (2020). Fe_3_O_4_ nanoparticles capped with PEG induce apoptosis in breast cancer AMJ13 cells via mitochondrial damage and reduction of NF-*κ*B translocation. *Journal of Inorganic and Organometallic Polymers and Materials*.

[69] Jabir M. S., Nayef U. M., Abdulkadhim W. K., Sulaiman G. M. (2019). Super magnetic Fe3O4-PEG nanoparticles combined with NIR LASER and alternating magnetic field as a potent anticancer agent against human ovarian cancer cells. *Materials Research Express*.

[70] Bahjat H. H., Ismail R. R., Sulaiman G. M. (2022). Photo detection properties of populated Fe3O4TiO2 core–shell/Si hetero junction prepared by laser ablation in water. *Applied Physics A*.

[71] Müller P., Ahmad M. (2011). Light-activated Cryptochrome Reacts with Molecular Oxygen to Form a Flavin–Superoxide Radical Pair Consistent with Magnetoreception. *J Biol. Chem.*.

